RETRACTED

# Application of Internet of Things Artificial Intelligence and Knowledge Innovation System in Table Tennis Teaching and Training

**DOI:** 10.1155/2022/7625626

**Published:** 2022-04-22

**Authors:** Yingmin Cui, Changlei Zhou

**Affiliations:** ^1^School of Physical Education, Hangzhou Normal University, Hangzhou, 311121 Zhejiang, China; ^2^College of Sports and Health, Linyi University, Linyi, 276000 Shandong, China; ^3^Department of Leisure Services and Sports, Pai Chai University, Daejeon Metropolitan City 35345, Republic of Korea

## Abstract

The Internet of Things is an important link in the future development of the Internet and will have a significant impact on development over the next five years or so. The purpose of this article is to learn how to use the Internet of Things to learn and practice table tennis and find new ways to integrate table tennis and the internet. This article proposes to build a detection system for IoT sensors and collect information about the ball's movement state and the athlete's movement state during table tennis. Through data analysis, we better guide athletes to develop table tennis training. At the same time, it also uses knowledge innovation to integrate the Internet of Things with the reality of life and better derive the development of the Internet of Things artificial intelligence. Based on this, this paper designs the construction of IoT sensors to collect the sports status of table tennis enthusiasts and verify the sports experience of table tennis enthusiasts by comparing factors such as physical training, basic skills and mobile training, interest, and confidence. The experimental results of this article show that the Internet of Things artificial intelligence has great potential, and it can innovatively promote industrial change. It better realizes the teaching and training of table tennis players and improves the teaching and training ability of table tennis by 20%.

## 1. Introduction

Table tennis is China's “national game.” China's table tennis performance in international competitions has always been ahead of other countries, occupying a dominant position in the world of table tennis. A large part of the reason is that table tennis is a traditional sport in China with a large mass base; at the same time, it is an advantageous project with mature technology and tactics and solid echelons at all levels. Because the operation of table tennis is simple and fast, and there is no special requirement for the body, men, women, and children all like table tennis. Table tennis is a sport full of skills and wisdom, which requires ever-changing skills and tactics, tenacious will, good thinking, and psychological qualities. Its peculiar sports characteristics play an important role in people's physical, mental exercise, and social adaptation. The knowledge innovation system is used in table tennis training to plan the development of table tennis as a whole and promote the technical upgrading of table tennis enthusiasts. At the moment when high technology is widely used in sports, table tennis has always stayed in the traditional confrontation training, which is not conducive to the improvement of table tennis, nor can it form a good table tennis teaching and training. How to better promote the innovative integration of the Internet of Things artificial intelligence in the teaching process of table tennis has become the focus of future work.

RETRACTED

For the innovative research of table tennis, experts and scholars at home and abroad have achieved a lot of results. Sève et al. study the action process of table tennis, focusing on how professional table tennis players mobilize knowledge related to their participation mode. Data is processed by transcribing the behavior and language expression of participants, decomposing their activities into basic meaning units, unit components, and identifying typical exploration and execution sequences. The results show that the knowledge that players mobilize in the game differs depending on the way they participate. Knowledge is constantly connected with important elements in the unfolding context to create a chain of interpretation, which helps to build a meaningful world [1]. Wu et al. work with data analysts to understand and describe the complex area of table tennis data analysis. They proposed a new interactive ping-pong program, iTTVis. It is the main visual analysis system for the analysis and analysis of table tennis data. ITTVis provides an overview of the entire game from the top three angles, creating a world of match analysis and calculation from a new perspective [2]. Leite et al. researched and investigated the game time structure in high-level table tennis matches to verify the influence of the evolution of international games on the game time structure. The duration of tension is the time required for long-term continuous training. The comparison between the three international events shows that the duration of the rally has been significantly reduced year by year, while the rest time has increased year by year. However, in the analysis of the competition stage, it was found that compared with the semifinals and finals, the rally duration of the quarter-finals was reduced, and the rest time increased from the quarter-finals to the semifinals and finals. It can be concluded that table tennis players need to take longer rest periods, and the evolution of the game and the stage of the game will affect the time structure of the table tennis game [3]. Bankosz and Winiarski conduct ping-pong kinematics, emphasize racket track trajectory, speed, and time characteristics, measure selected ping-pong kinematics during before and after shifts, and design rifle variations. At the same moment, the study included 12 female ping-pong athletes who practiced high-performance sports and performance. Each keyword must complete a series of six tasks and enter different types of topspin. *Result*: the largest racket trajectory is related to the forehand, counterspin and winning ball [4]. Ngo et al. evaluate the performance of table tennis synchronization with physiological and motor subject variables. Nine table tennis players completed a series of low- and high-stress services with the team's crossover design. An automated animation system with a high-speed 3D motion camera and an animator determines the dynamics of an object: bats, angles, and timers. The angle of the bat's face refers to the different angles presented by subjects moving in different directions like a bat. Reported heart rate status and measurements were collected to assess changes in various conditions. Contrary to popular belief, the angle of a bat's face does not change significantly in a state of anxiety. In the most frightening situations, bats move faster [5]. Yoichi et al. investigate the mechanical power generation of the paddle arm and the principle of transmission of the table tennis arm. Ten male table tennis players using their right hand use the top rotation to get rid of the top rotation and the back rotation. The inverse kinetics method was used to measure the joint function of the paddle shoulder, elbow, and wrist. Inverse dynamics is a branch of mechanics. It is a bridge that connects dynamics and kinematics. It indirectly determines the process of force and moment according to the kinematics and inertial characteristics of the moving human body. It is concluded that during the forward swing, most of the mechanical energy obtained by the racket arm comes from the energy transfer of the torso. Shoulder joint vertical energy transfer of force is the largest factor of mechanical energy of the mela arm into two bends and larger at the opposite bend than at the upper bend [6]. Wang et al. proposed a hybrid Markov chain model for adults to describe and simulate table tennis tournaments, along with Tac Simur's imaging system to create visual analysis simulations. The Markov chain is a random process that features Markov properties in mathematics. In this process, based on current knowledge or information, the past (i.e., the historical situation of the present) is not involved in predicting the future (i.e., the state of the future after the present). Tac Simur allows users to guide different players and their techniques according to their in-game practices to determine which players and techniques are interested in further analysis [7]. The study of Meghdadi et al. examined the time difference and intensity of shoulder muscle activity between table tennis players with and without shoulder shock symptoms during arm rotation, by measuring the timing and level of activity of the lower rectangular spine and the anterior serratus, the anterior shoulder muscle, the supraspinatus muscle, and the biceps muscle of 30 healthy players. As a result, the order of activation and selection of shoulder muscles in people with shock symptoms changes, suggesting that shock symptoms may be associated with shoulder muscle dysfunction [8].

RETRACTED

Based on the application of artificial intelligence in the Internet of Things, this article innovatively proposes a method of upgrading the teaching and training mode of table tennis. The advantages are as follows: (1) through the construction of the Internet of Things detection and evaluation analysis system, comprehensive analysis of table tennis related data, and formulation of optimal strategies, (2) finding a measure of the certainty of table tennis technology to better determine the training effect, and (3) the questionnaire was designed to lead the experiment before and after the experiment, to better understand the changes in interest and confidence of table tennis enthusiasts before and after training.

## 2. Internet of Things Artificial Intelligence Innovation Method

### 2.1. Internet of Things

The Internet of Things is also called a network of sensors. It is distributed according to the traditional architecture of the Internet of Things [9]. The Internet of Things can be divided into intellectual layers, network layers, and application layers, as shown in Figure 1.

1. Perception layer

The identification layer underlies the three-tier system architecture of the Internet of Things and is the source of information for the Internet of Things. As the name suggests, the identification layer is used primarily to specify information about objects. The Internet of Things is the web of everything, and information about things is the foundation of the Internet of Things. Detector layer is a network of various sensors, and the actual IoT system has many sensors such as temperature and humidity camera, light, smoke, and pressure sensor. The protocols used by the sensors are also different, such as wireless personal area network, wireless LAN, and remote computer interface protocol. At present, many IoT systems use customized sensors, customized communication protocols, and system specificity.

(2) Network layer

The network layer is a connecting layer in the three-tier architecture of the Internet of Things, the sensor access is managed through technologies such as the Internet of Things gateway, and the collected data is reliably and stably transmitted to the application layer. There are also many communication protocols at the network layer, such as mobile Internet, mobile communication networks, wireless sensor networks, and wired and wireless local area network, and sometimes private networks are used for transmission. The network layer not only has to deal with complex sensor communication protocols but also uses different protocols to interact with the application layer. Professionals with knowledge of network communication are often required for design and management.

(3) Application layer

The application layer is located at the top of the three-tier architecture system of the Internet of Things and is the embodiment of the application of the Internet of Things system. No matter how complex the IoT system is, in the final analysis, specific applications must be formed to have value. The application layer analyzes and processes the data transmitted by the network layer and stores and displays the results. According to the functions and use, IoT applications can be found in different industries, such as industry, medical care, environment, safety, and transportation, with a wide range of applications and multiple disciplines. Therefore, the Internet of Things system presents the characteristics of very different functional styles and strong professionalism.

RETRACTED

### 2.2. Artificial Intelligence

Artificial intelligence is a technology developed based on a combination of disciplines based on artificial neural networks [10]. In the research of the artificial nervous system, the main topic is analysis, and its flexibility is achieved through analysis. During the learning process, the weight of the connection is adjusted according to some changes in the environment to improve the behavior of the system to achieve the goal. The artificial nervous system has the properties of large-scale parallel processing and distributed storage, as well as the ability to adapt and design. It features classification and identification and improves calculations and nonmapping linear. Artificial neural systems include a variety of species such as BP, Hopfield feedback, SOM (self-organizing mapping) properties, and CPN dual distribution of neural networks [11]. The structure is shown in Figure 2. The Hopfield neural network is a recurring neural network, which is a neural network that connects storage systems and two systems. This results in a combination with the local minimum, but the combination with the local minimum is wrong and may also have a global minimum. The Hopfield network also offers models that mimic smaller models. Self-regulatory property mapping is a competitive network study that can identify “near and remote voltage blocking” activity in the nervous system of the brain by competing between neurons and can map input at low dimensions. CPN was first used to implement a sample selection matching system. CPN networks can store binary or analog pattern pairs, so this network model can also be used for associative storage, pattern classification, function approximation, statistical analysis, and data compression.

RETRACTED

The BP neural network is considered to be the most common and successful neural network, and its structure is shown in Figure 2. The propagation of forward signals and the spread of backward errors form the BP neural network analysis process. As the signal continues to propagate, the data flows from the input layer to the hidden layer and eventually to the output layer. The actual return on the conversion layer is compared with the expected value. If it does not match, it goes to the error recovery phase. At this point the resulting error is returned to the input layer by layer hidden in one form or another. All the neurons in each layer share the error, take the error signal from each layer of the nerve cell, and change the weight of each nerve cell based on that signal. During the learning process of the network, the weights will be adjusted until the end of the training. Among them, in the field of mathematics, weight refers to the frequency of each number in the weighted average, also known as weight or weight. Whether the learning process ends depends on the network output error and the number of learning times, and it ends when the output error or learning times of the network meet the conditions [12].

It can be seen from Figure 3 that the BP neural network is composed of an input layer, an output layer, and an intermediate layer (or hidden layer). Among them, *a*_*x*_ represents the input of the neural network, *b*_*x*_ represents the actual output of the neural network, and *c*_*x*_ represents the expected output of the neural network; *Q*_*mef*_ represents the connection weight of the *e*th neuron of the *m*th layer to the *f*th neuron of the *m* + 1th layer; *S*_*me*_ represents the output of the *e*th neuron in the *m*th layer; *Y*_*me*_ represents the threshold of the *e*th neuron in the *m*th layer, and among them, the threshold is also called the critical value, which refers to the lowest or highest value that an effect can produce; *Z*_*me*_ is expressed as the total input of the eth neuron in the *m*th layer; *J*_*m*_ represents the number of neurons in the *m*th layer. The above figure is an example to derive the standard BP algorithm.

RETRACTED

As described below, ① forward propagation calculation is as follows:

(1) $$\begin{array}{c} Z_{me}=\overset{J_{m-1}}{\underset{f=1}{\sum }}S_{\left(m-1\right)f}*Q_{\left(m-1\right)fe},\\ Q_{me}=f_{s}\left(Z_{me}\right)=\frac{1}{1+\exp\left[-\left(Z_{me}-Y_{me}\right)\right]}. \end{array}$$

② Return algorithm means that the input function proceeds level by layer from the input level to the hidden level and then to the output level. The location of each level of neurons only affects the location of the next layer of neurons. If neuron *e* is in the output layer, then *S*_*me*_ is the actual output, and record it as according to *b*_e_; the error generated by and the expected output *c*_*e*_ are backpropagated to modify the weights. The error definition can be expressed by the following formula (2):

(2) $$\begin{array}{c} b_{\text{e}}w_{\text{e}}=c_{e}-b_{e}. \end{array}$$

The network objective function can be expressed as follows:

(3) $$\begin{array}{c} I=\frac{1}{2}\underset{e}{\sum }{\left(c_{e}-b_{e}\right)}^{2}. \end{array}$$

The weights are corrected in the direction of the gradient drop of the *I* function, as follows:

(4) $$\begin{array}{c} \Delta Q_{mef}=-\lambda \frac{\partial I}{\partial q_{mef}}. \end{array}$$

Among them, 0 < *λ* < 1 is learning efficiency.

If it will want to program directly to calculate this, it must calculate the recurrence relationship between *q* and neuron output, as described below:

(5) $$\begin{array}{c} \Delta Q_{mef}=-\lambda \frac{\partial I}{\partial q_{mef}}=-\lambda \frac{\partial Q}{\partial Z_{\left(m+1\right)f}}*\frac{\partial Z_{\left(m+1\right)f}}{\partial q_{mef}}={\lambda \theta }_{mf}\frac{\partial Z_{\left(m+1\right)f}}{\partial q_{mef}}. \end{array}$$

In

(6) $$\begin{array}{c} \theta_{mf}=-\frac{\partial I}{\partial Z_{\left(m+1\right)}f},\\ \frac{\partial Z_{\left(m+1\right)f}}{\partial q_{mef}}=\frac{\partial }{\partial q_{mef}}\left(\sum S_{md}*Q_{mcf}\right)=S_{mf},\\ \Delta Q_{mef}=-\lambda \frac{\partial I}{\partial q_{mef}}=-{\lambda \theta }_{mf}S_{me},\\ \theta_{mf}=-\frac{\partial I}{\partial Z_{\left(m+1\right)f}}=-\frac{\partial I}{\partial S_{\left(m+1\right)f}}*\frac{\partial S_{\left(m+1\right)f}}{\partial Z_{\left(m+1\right)f}}. \end{array}$$

Make

(7) $$\begin{array}{c} \frac{\partial S_{\left(m+1\right)f}}{\partial Z_{\left(m+1\right)f}}=f^{\prime }\left(Z_{\left(m+1\right)f}\right),\\ f^{\prime }\left(x\right)=\frac{e^{-\left(x-f^{..}\right)}}{{\left[1+e^{-\left(x-f^{..}\right)}\right]}^{2}}=f\left(x\right)\left[1-f\left(x\right)\right],\partial I/\partial S_{\left(m+1\right)f}S_{\left(m+1\right)f}\frac{\partial I}{\partial S_{\left(m+1\right)f}}=b_{f}-c_{f},\theta_{mf}=-\frac{\partial I}{\partial Z_{\left(m+1\right)f}}=-\frac{\partial I}{\partial S_{\left(m+1\right)f}}*\frac{\partial S_{\left(m+1\right)f}}{\partial Z_{\left(m+1\right)f}}=\left(c_{f}-b_{f}\right)S_{\left(m+1\right)f}\left(1-S_{\left(m+1\right)f}\right),\frac{\partial S_{\left(m+1\right)f}}{\partial Z_{\left(m+1\right)f}}=f^{\prime }\left(Z_{\left(m+1\right)f}\right)=f\left(Z_{\left(m+1\right)f}\right)\left(1-f\right)=S_{\left(m+1\right)f}\left(1-S_{\left(m+1\right)f}\right). \end{array}$$

Discuss the classification of, *∂I*/*∂S*_(*m* + 1)*f*_ and when *S*_(*m* + 1)*f*_ is the output node,

(8) $$\begin{array}{c} \frac{\partial I}{\partial S_{\left(m+1\right)f}}=b_{f}-c_{f},\\ \theta_{mf}=-\frac{\partial I}{\partial Z_{\left(m+1\right)f}}=-\frac{\partial I}{\partial S_{\left(m+1\right)f}}*\frac{\partial S_{\left(m+1\right)f}}{\partial Z_{\left(m+1\right)f}}=\left(c_{f}-b_{f}\right)S_{\left(m+1\right)f}\left(1-S_{\left(m+1\right)f}\right),\\ \theta_{mf}=\left(c_{f}-b_{f}\right)b_{f}=\left(c_{f}-S_{nf}\right)S_{nf}\left(1-S_{nf}\right). \end{array}$$

When *S*_(*m* + 1)*f*_ is a hidden node, then

(9) $$\begin{array}{c} \frac{\partial I}{\partial S_{\left(m+1\right)f}}=\overset{J_{m+1}}{\underset{g=1}{\sum }}\frac{\partial I}{\partial Z_{\left(m+2\right)g}}*\frac{\partial Z_{\left(m+2\right)g}}{\partial S_{\left(m+1\right)f}}=-\overset{J_{m+2}}{\underset{g=1}{\sum }}\theta_{\left(m+1\right)g}q_{\left(m+1\right)fg},\\ S_{me}=\overset{J_{m+2}}{\underset{f=1}{\sum }}S_{\left(m-1\right)f}*q_{\left(m-1\right)fe}. \end{array}$$

For *S*_(*m* + 1)*f*_, when it belongs to a hidden node, the actual output of the point can be known, but the correct output cannot be known in advance. The total error is closely related to the output of the hidden layer, and the output of this layer can affect the output of all nodes in the next layer.

(10) $$\begin{array}{c} \theta_{mf}=S_{\left(m+1\right)f}\left(1-S_{\left(m+1\right)f}\right)\overset{J_{m+2}}{\underset{g=1}{\sum }}\theta_{\left(m+1\right)g}q_{\left(m+1\right)fg}. \end{array}$$

The weight adjustment formula of this algorithm can be expressed as follows:

(11) $$\begin{array}{c} \Delta Q_{mef}=\left\{\begin{array}{c} \lambda \left(c_{f}-b_{f}\right)b_{f}\left(1-b_{f}\right)S_{me},m+1m+1\text{ is the input layer},\\ \lambda S_{\left(m+1\right)f}\left(1-S_{\left(m+1\right)f}\right)\left(\overset{J_{m+2}}{\underset{g=1}{\sum }}\theta_{\left(m+1\right)g}q_{\left(m+1\right)fg}\right)S_{me},m+1\text{ is the hidden layer}. \end{array}\right. \end{array}$$

The neurons in the mth layer can be expressed as follows:

(12) $$\begin{array}{c} S_{mf}=\left\{\begin{array}{c} \left(c_{f}-b_{f}\right)b_{f}\left(1-b_{f}\right),m+1m+1\text{ is the input layer},\\ S_{\left(m+1\right)f}\left(1-S_{\left(m+1\right)f}\right)\left(\overset{J_{m+2}}{\underset{g=1}{\sum }}\theta_{\left(m+1\right)g}q_{\left(m+1\right)fg}\right),m+1\text{ is the hidden layer}, \end{array}\right.\\ Q_{mef}\left(r+1\right)=Q_{mef}\left(r\right)+\Delta Q_{mef}=Q_{mef}+{\lambda \theta }_{mf}S_{me}. \end{array}$$

The same proof is as follows:

(13) $$\begin{array}{c} \Delta \theta_{mf}=-\lambda \frac{\partial I}{\partial \theta_{mf}}=\left\{\begin{array}{c} \lambda \left(c_{f}-b_{f}\right)b_{f}\left(1-b_{f}\right),m+1m+1\text{ is the input layer},\\ \lambda S_{\left(m+1\right)f}\left(1-S_{\left(m+1\right)f}\right)\left(\overset{J_{m+2}}{\underset{g=1}{\sum }}\theta_{\left(m+1\right)g}q_{\left(m+1\right)fg}\right),m+1\text{ is the hidden layer}. \end{array}\right. \end{array}$$

RETRACTED

### 2.3. Knowledge Innovation

For knowledge, the explanation given by the modern Chinese dictionary is as follows: knowledge is the generalization of experience and knowledge gained by the masses in the actual work of reforming the reality. In the process of analyzing knowledge-related concepts, Chinese scholars and Western scholars have reached a consensus on the classification of knowledge, that is, knowledge is divided into explicit knowledge and tacit knowledge [13]. Explicit knowledge, also known as textable knowledge, can be expressed with the help of standards and overall language, making the process of dissemination, communication, and sharing more convenient, and it is the information that people can use comprehensively; tacit knowledge includes beliefs, metaphors, intuitions, thinking patterns, and so-called “knowledges,” and it is a kind of tacit understanding between people, which is formed through continuous running-in in the complex market structure, and has the characteristics of being difficult to express and highly individualized.

Knowledge innovation is a dynamic process, which consists of knowledge creation, evolution, transfer, and application. Among them, the creation of knowledge refers to the creation of new knowledge on the basis of predecessors, the evolution of knowledge is the process of gradually enriching and perfecting knowledge theory, and the transfer of knowledge is the process of applying knowledge to other fields, and the application of knowledge refers to the process of transforming knowledge achievements. It relies on the discovery of new laws, the exploration of new discoveries, and the accumulation of new knowledge to achieve the goal of completing individual, overall, and unit competitive advantages and increasing the added value of knowledge [14]. For the concept of knowledge innovation, there are broad and narrow definitions in general. Knowledge innovation in a broad sense, the specific content involved is follows: knowledge, mechanisms, systems, management, technology, thought, operation, and other innovations that can create value. In the narrow sense, knowledge innovation distinguishes knowledge innovation from management innovation and technological innovation and conducts research only on knowledge innovation led by scientific research. Knowledge innovation is a system. The knowledge innovation system is a network system composed of institutions and organizations related to the production, diffusion, and transfer of knowledge. The structure is shown in Figure 4. The national knowledge innovation system is the foundation and engine for cultivating and driving the development of the knowledge economy. The knowledge innovation system not only includes technological innovation but also includes organizational innovation, management innovation, and institutional innovation [15]. The origin of the structure refers to the application of knowledge and methods of behavioral science. It combines the expectations of human growth and development with organizational spaces, and through reforms and changes in the organizational structure and management systems, it can adapt to changes in the external and internal environment of the organization, thus improving the efficiency of activities. Management certification refers to the creation of creative, noncreative, funds, information, power, and other components of the system through scheduling, scheduling, authorization, integration, management, feedback, and other media over a period of time conditions, to meet the new demands of human activities of biological flow, unnatural flow, capital flow, information flow, and energy flow. Industrial innovation is a prerequisite for innovation, and a complete business system optimization system can ensure the effective advancement of technological innovation and management innovation.

RETRACTED

### 2.4. The Development Status of Table Tennis

According to relevant research findings, there are nearly 150 million enthusiasts in China who regularly participate in table tennis. Participants have a certain proportion of men, women, and children, and the age span is very wide. Among them, young ping-pong enthusiasts account for about 20% of the total number, which can be as high as 30 million. Young ping-pong enthusiasts use table tennis as a sports activity in their spare time, which can achieve the purpose of strengthening their bodies and invigorating their bodies and minds. Although table tennis does not require high physical fitness, the diversity and complexity of its sports technology has higher requirements for the training of young table tennis enthusiasts [16]. Therefore, in the context of this research, it is essential to design a training program for table tennis enthusiasts.

The training and teaching of table tennis is based on physical training, the technology is based on basic skills and mobile training, and the focus is on the coach's tactical training. Among them, physical training refers to training such as footwork and endurance, and basic skills and movement training refer to related technical operations such as the technique of serving and receiving the ball. Unfortunately, the number of trainers with professional knowledge cannot match the increasing number of table tennis enthusiasts.  Figure 5 shows the coaches instructing teenagers to practice ball. In this case, it is particularly important to use portable and simulated guidance methods for professional coaches to carry out effective and reasonable sports training. With the continuous research and development of smart wearable devices and the wide application in the field of sports training, it has directly promoted the role of big data in the field of sports training [17]. Through the extensive collection, storage, and application of various index parameters of athletes' training in the early, mid, and late stages of training, the information resources that coaches can use have been greatly enriched, and it also improves the objectivity of coaches for quantitative evaluation of athletes' sports performance feedback and adds new vitality to sports training. As a typical representative of emerging smart products in the era of big data, sensors are multidisciplinary cutting-edge technology products developed from microelectromechanical systems based on microelectronics technology. They have small size, light weight, low power consumption, high reliability and sensitivity, low price, and other advantages [18]. The table tennis sensor used in this research is a very universal sensor product designed by combining an accelerator, a gyroscope, and a magnetometer, as shown in Figure 6. The rational use of smart table tennis sensors in the exercise of traditional table tennis techniques can greatly improve the efficiency of training, and it can also allow coaches to construct teaching methods and training methods that combine big data to raise the goal of scientific training to a new level [19].

RETRACTED

## 3. Table Tennis Teaching and Training Experiment and Analysis

### 3.1. Object

The practical application of smart table tennis sensor to the amateur table tennis training of teenagers and children is the research object. Survey object is:80 amateur tennis students from the table tennis club, aged 10-60, with more than half a year of tennis experience and able to participate in training for more than three times a week. The details are shown in Table 1.

### 3.2. Methods

1. Document method

Comprehensively understanding the training status of amateur table tennis players, analyze their problems in the training process, and explore the application of intelligent sensors in the field of sports. Through the Wanfang database and CNKI, we have consulted and collected research literature on amateur table tennis training, smart sensors, and smart wearable devices to understand the research and development process related to this topic. Using scientific and reasonable methods, the classification, analysis, and summary of related documents were carefully carried out, which laid a solid foundation for the writing of this paper [20].

(2) Expert interview method

To enhance the reliability and feasibility of this practical research, we consulted many coaches and teachers with rich experience and achievements in the field of sports training through interviews, interviews, telephone interviews, etc. Among them, there are 2 professors and 4 associate professors. Experts have put forward many valuable opinions and suggestions for this study, and they also give unique views on the impact of smart table tennis, sensors on table tennis training, and the impact of equipment on table tennis training in the future. Experts in the design of the experimental ideas and questionnaire content of this practical research all expressed their approval and pointed out the direction of this research.

(3) Questionnaire survey method

The table tennis learning interest questionnaire is designed by consulting the relevant literature and materials of this practical research and combining with the previous training experience in the club, which mainly aimed at amateur table tennis enthusiasts after using smart table tennis sensors to investigate and study the value of table tennis sports. Before using the smart table tennis sensor, a total of 80 questionnaires were distributed to the trainees participating in this practical training in the form of on-site questionnaires. 80 questionnaires were returned after filling in the field, and 80 questionnaires were effectively returned. After using the smart table tennis sensor, 80 questionnaires were distributed to the trainees participating in this practical training, and 80 questionnaires were effectively collected. To make the content of the questionnaire of this practical research consistent with the research purpose, 9 experts were specifically asked to evaluate the validity of the questionnaire of this practical research. Among them, 6 experts thought that the content of the questionnaire was perfect, accounting for 66.7% of the total number of people, and the remaining 3 experts said that the content of the questionnaire was relatively perfect. The overall recognition rate is 100%. The content of the questionnaire is shown in Table 2.

RETRACTED

It can be seen from Table 2 that the value of smart sensors has been recognized by most people, but there are still some people who do not recognize the effects of smart sensors. Based on the above survey results, coaches can formulate targeted solutions to help athletes formally recognize and reasonably use smart sensors.

### 3.3. Experimental Method

Using the same training plan for group training, and the training time is two months. The training content is based on basic physical training, forehand attacking, backhand attacking, receiving and serving, left push and right attack, and other basic skills, multiball training, etc., as the teaching content. The training effects of the experimental group and the control group are compared and analyzed based on the results of the international training test. Through the overall measurement of the impact of athletes on improving the stability of the batting action, standardizing basic technical movements, improving the ball feel, etc., it is verified whether the use of smart table tennis sensors and its supporting applications to assist training can effectively improve the efficiency of training and produce actual results.

### 3.4. Experimental Design

The 80 table tennis enthusiasts all have 8 weeks of basic table tennis technical and physical training, the first 3 weeks are basic training, and the last 5 weeks are intensive training. The experiment is divided into two groups on average, and the corresponding ratios of each age group are drawn to form a speed measurement group. The experimental group wears smart sensors, and the control group remains the same. The training frequency is 3 times a week (24 hours apart), and each class is trained for 90 minutes. Each coach is one-to-three to ensure that the training duration of each student is the same, and other standards remain the same. The specific training plan in the early stage is shown in Table 3. The plan is formulated after discussion and communication by many experts.

RETRACTED

To ensure the fairness of the experiment, the coach is only responsible for explaining the training content and will not answer questions from the tester during and after the training. In addition, all testers are not allowed to practice after the training. The experimental group used smart table tennis, sensors, and supporting APPs in the process of participating in training. During training, some technical indicators of the participants in the experimental group can be connected to the APP through the smart table tennis sensor and reflected in the APP, such as average racquet speed and number of swings. And complete the training according to the basic physical and technical training courses that the APP comes with. And combine with the ranking function in the APP discussed in the WeChat group. Participants in the control group only participated in the training and did not use table tennis, smart sensors, and supporting APPs. The discussion in the WeChat group was not based on technical indicators. The training results are shown in Figure 7.

It can be seen from Figure 7 that the various abilities of the trained athletes have been improved to a certain extent. Compared with the control group, the test group's data performs well, but in general, the overall difference is not big. It shows that there is little difference in basic training with or without sensors in a short period of time.

After the first stage of training is over, start the second stage of training. The second stage includes a five-week training program, mainly in skills, techniques, and multiball training. The specific course schedule is shown in Table 4.

It can be seen from Figure 8 that in the same venue, the same amount of training time, and the same level of starting point, this fully shows that the smart table tennis sensor has a good effect in daily teaching and training. On the basis of auxiliary daily training, it also stimulated the active curiosity of table tennis students to practice more actively and achieve better results. After training, the athletes basically mastered table tennis techniques, and the performance of the test group and the control group improved. Compared with the control group, the test group has a greater improvement in performance, and overall, the improvement effect is better. The speed test results showed significant differences.

It can be seen from Figure 9 that after the operators have been trained, various indicators have risen, especially the standardization of movements and technical stability have been greatly improved, and the test group has the largest improvement. Relatively stable physical fitness improved, but there was little difference between the test group and the control group, which should require longer exercise. To compare and analyze the reasons for the difference in data between the two, the sensors in the test group also receive various data from the athletes to form a promotion curve. Athletes can perform targeted exercises based on the promotion curve of their own data to improve their abilities. At the same time, based on the athlete's own data, the coach can also carry out personalized training based on the data to train each athlete to become a talent. Through the summary function of the intelligent table tennis training system platform, the workload of the “coach” is reduced, and the time occupied by the subjects of the experimental group is reduced. The biggest advantage is that the platform system has a cloud storage function to ensure data security and enables trainers to query the subjects' exercise data anytime and anywhere, which is convenient for management.

RETRACTED

After the experiment, we investigated the athletes' psychological feelings after training. With reference to the opinions of experts, a questionnaire on interest and confidence in table tennis was developed to evaluate athletes' psychological status from three indicators: very suitable, basically suitable, and inappropriate. Compare the questionnaire survey before the experiment to ensure the reliability of the questionnaire. The questionnaires are distributed face to face and filled in face to face. If there are any questions, it can communicate with each other to ensure the authenticity and accuracy of the content and ensure that there are no invalid questionnaires. The return rate of the two rounds of questionnaires was 100%. The result is shown in Figure 10.

From the results in Figure 10, it can be seen that the use of smart table tennis sensors and its supporting APPs to assist table tennis training deepens the user's interest in table tennis. On the one hand, it is because the product itself visualizes and concretizes the technical movements of table tennis; on the other hand, it is through the technical data of the experimental group of students' swing speed and the number of swings collected in the APP that allow students to intuitively see the gap with those around them. This fully mobilized the subjective initiative of the experimental group of students to actively participate in the training, thereby deepening their interest in table tennis and improving the training effect. According to the statistical data of the sports confidence of the two groups of students before and after the experiment, it can be seen that after the practical training, the athletes' lack of confidence has greatly decreased. From this, we can see that the improvement of ability and other aspects will increase confidence.

RETRACTED

## 4. Discussion

By observing the difference in the structure of table tennis training between the experimental group and the control group before and after the experiment, it can be seen that after the experimental group of students uses smart table tennis sensors to assist in training, their scores on various indicators such as physical fitness, technology, and specification are significantly better than those of the control group. The difference in the test data of the two groups of students is significant, which verifies the effect of the experimental design. Data were collected using smart table tennis sensors on various techniques of the experimental group of students before and after training using the smart table tennis sensors to assist training. Through the difference analysis, it can be known that the difference of the various technical data of the experimental group of students before and after the training is highly significant. This also verifies that the use of smart tennis sensors to assist amateur table tennis students in training is feasible and can improve training efficiency, and it can also have a positive impact on training. Through the curves and graphs of the interest and confidence of table tennis enthusiasts, it can be clearly seen that the sensor has important guiding significance to enhance the interest of table tennis enthusiasts and can better enhance the confidence of table tennis enthusiasts. In the future, the integration of table tennis and sensors should be better promoted to guide the improvement of table tennis enthusiasts.

## 5. Conclusions

This article conducts research on table tennis training and teaching and monitors the training process of table tennis with the help of Internet of Things and new artificial intelligence sensors. Measuring the relevant indicators of athletes and compare them to athletes who do not use sensors. Sensors can increase interest and confidence in table tennis and improve athletes' various skills. To a certain extent, it can also reduce the burden on the coach. In general, the application of sensors can better understand the development of table tennis and meet the needs of the masses for improving table tennis skills. However, the sensor also has the following shortcomings. In the process of measurement, there may be inaccurate data due to the capture efficiency of the sensor. The stability of the Bluetooth connection is insufficient, and the device may be disconnected when used with the mobile phone supporting software. The comfort of equipment installation is insufficient, and the cost is not low. In the future, we will further improve the deficiency and increase related investment, so that more sensors can be used in table tennis teaching and help table tennis enthusiasts improve their level.

RETRACTED

## Figures and Tables

**Figure 1:** The three-tier structure of the Internet of Things.

**Figure 2:** Schematic diagram of artificial neural network structure.

**Figure 3:** Schematic diagram of BP neural network structure.

**Figure 4:** National knowledge innovation system structure.

**Figure 5:** Coaches instruct young people to practice table tennis.

**Figure 6:** Schematic diagram of the structure of the table tennis sensor.

**Figure 7:** Comparison of basic indicators between the test group and the control group before and after the experiment.

**Figure 8:** Comparison of various values between the test group and the control group training.

**Figure 9:** Comparison of various indicators before and after the athletes' training.

**Figure 10:** Comparison of interest and self-confidence of athletes before and after the experiment.

**Table 1:** Age composition of table tennis players.

	10-18		18-25		25-40		40-60	
Total (person)	30	5	26	9	5	3	1	1
Training time (year)	Half a year	One year	Half a year	One year	Half a year	One year	Half a year	One year

**Table 2:** Questionnaire on the use value of table tennis sensors.

	Yes	No	Other
Do you think smart table tennis sensors are helpful for you to improve your exercise norms?	60%	8.5%	31.5%
Teaching through smart ping-pong sensors whether you are motivated to learn independently	72%	4.7%	23.3%
Compared with traditional teaching methods, do you think that smart table tennis sensor teaching is more superior?	68%	3.9%	28.1%
Do you improve your deep understanding of technical concepts through smart table tennis sensor teaching?	71%	5.1%	23.9%
Does the smart table tennis sensor improve your ability to find and solve technical problems?	77%	2.3%	20.7%

**Table 3:** The first stage training plan of athletes.

Training time	Training course	Training content
The first week	Basic physical training	Speed training
		Endurance training
		Strength training

The second week	Basic skill training	Action training
		Style shaping and technical shaping training.

The third week	Mobile training	Anticross step
		Positive cross step
		Movement speed training

**Table 4:** Course schedule for the second stage.

Training time	Training course	Training content
The fourth week	Forehand serve	Forehand serve
		Forehand turning and nonturning
		High forehand serve

The fifth week	Backhand serve	Backhand fast and fast backspin
		Right backhand up (down) spin

The sixth week	Push offense	Push left and attack right
		Left push combined with backhand attack

The seventh week	Rubbing	Forehand and backhand rubbing combined with forehand quick pull, hurry up, assault, or smash
		Forehand and backhand rubbing combined with backhand quick pull, hurry up, assault, or smash

The eighth week	Two-sided attack	Tap left and buckle right
		Attack the two corners, slam into the middle

RETRACTED

## Data Availability

All the data used is given in the paper.
